# InSilc Computational Tool for *In Silico* Optimization of Drug-Eluting Bioresorbable Vascular Scaffolds

**DOI:** 10.1155/2022/5311208

**Published:** 2022-09-05

**Authors:** Miljan Milosevic, Milos Anic, Dalibor Nikolic, Bogdan Milicevic, Milos Kojic, Nenad Filipovic

**Affiliations:** ^1^Bioengineering Research and Development Center, BioIRC, Kragujevac, Serbia; ^2^Institute for Information Technologies, University of Kragujevac, Kragujevac, Serbia; ^3^Belgrade Metropolitan University, Belgrade, Serbia; ^4^Faculty of Engineering, University of Kragujevac, Kragujevac, Serbia; ^5^Houston Methodist Research Institute, Department of Nanomedicine, Houston, USA; ^6^Serbian Academy of Sciences and Arts, Belgrade, Serbia

## Abstract

Stents made by different manufacturers must meet the requirements of standard *in vitro* mechanical tests performed under different physiological conditions in order to be validated. In addition to *in vitro* research, there is a need for *in silico* numerical simulations that can help during the stent prototyping phase. *In silico* simulations have the ability to give the same stent responses as well as the potential to reduce costs and time needed to carry out experimental tests. The goal of this paper is to show the achievements of the computational platform created as a result of the EU-funded project InSilc, used for numerical testing of most standard tests for validation of preproduction bioresorbable vascular scaffolds (BVSs). Within the platform, an ad hoc simulation protocol has been developed based on the finite element (FE) analysis program PAK and user interface software CAD Field and Solid. Two different designs of two different stents have been numerically simulated using this integrated tool, and the results have been demonstrated. The following standard tests have been performed: longitudinal tensile strength, local compression, kinking, and flex 1-3. Strut thickness and additional pocket holes (slots) in two different scaffolds have been used as representative parameters for comparing the mechanical characteristics of the stents (AB-BVS vs. AB-BVS-thinner and PLLA-prot vs. PLLA-plot-slot). The AB-BVS-thinner prototype shows better overall stress distribution than the AB-BVS, while the PLLA-prot shows better overall stress distribution in comparison to the PLLA-plot-slot. In all cases, the values of the maximum effective stresses are below 220 MPa—the value obtained by *in vitro* experiment. Despite the presented results, additional considerations should be included before the proposed software can be used as a validation tool for stent prototyping.

## 1. Introduction

Drug-eluting balloon-expandable stents are commonly used to treat coronary lesions in the process of percutaneous transluminal coronary angioplasty (PTCA) [1]. PTCA has been shown to have some disadvantages such as potential inflammation, late-stent thrombosis, neoatherosclerosis, and restenosis [2–4]. To overcome some of the shortcomings, bioresorbable vascular scaffolds (BVSs) were introduced [5, 6]. The basic idea is to use BVSs as temporary scaffolds in the first 6-12 months after PTCA. The degradation of a BVS usually takes place 12 to 24 months after PTCA, while their disappearance from the human body occurs after 36 months [7]. BVSs are mainly built using bioresorbable polymers and biocorrosive metal alloys, covered by biodegradable drug-eluting polymers. Stents with biodegradable coatings are usually named “partially BVS” while stents with a biodegradable backbone material are indicated as “fully BVS” (or also as a bioresorbable scaffold, BRS). Bioresorbable polymers are generally a hundred times softer compared to biocorrosive metal alloys [8] while biocorrosive metal alloys have an unpredictable degradation rate. The softness of bioresorbable polymers can cause serious complications due to significant recoil, early or late [9–11]. In contrast, the unpredictable biodegradability of biocorrosive metal alloys increases the risk for thrombosis and restenosis [12]. Despite the advantages and disadvantages of both materials, it was shown in [13] that bioresorbable polymers are the better choice. Therefore, additional research was performed in the past to analyze the impact of stent geometry change on recoil reduction in bioresorbable scaffolds. For example, in [14], it was shown that the rates of radial and longitudinal recoil and the rates of dog boning are mostly affected by geometry, artery surface ratio, and stent strut thickness.

Each manufacturer must meet the ISO standard and validate the stent prototype using standard mechanical tests. Since these tests are usually very expensive and time-consuming, there is a need for *in silico* tests based on computational numerical simulations. However, for *in silico* tests to be used, it is necessary to develop sufficiently accurate, robust, and applicable material models and also to validate the approach by comparing it with the experiment. Among the computational methods, the finite element method (FEM) is mainly used for stent analysis. The FEM has so far proven to be the method of choice in the prediction of structure degradation during cyclic loading [14] or for the construction of new material models [15–19]. A lot of effort has been made in the past to create an adequate material model for biodegradable stents. These material models are mainly based on hyperelastic and viscoplastic behavior [12] and generally require a large number of material parameters [20]. A model involving the influence of a strain rate and kinematic/isotropic hardening was introduced in [13, 21]. In [22], a new material model for biodegradable polymeric PLLA scaffolds, based on the direct use of experimentally obtained uniaxial tensile stretch-stress curves, was introduced. This material model does not require a usually large number of material parameters evaluated by fitting procedure with experiments, so it can be easily applied with a satisfactory representation of biodegradable materials. The main advantage of the model is that the input can be any multilinear curve obtained from the manufacturer.

The material model presented in [22] was a result of the InSilc project whose goal was to develop a finite element- (FE-) based methodology for modeling coronary drug-eluting bioresorbable vessel scaffolds (BVSs). It was shown in [22], by validating and comparing with an experiment, that such methodology can mimic *in vitro* inflation, radial compression, and crush resistance mechanical tests for partially BVS device (SYNERGY™ BP) and a prototype bioresorbable stent (PLLA-prot). In [23], we demonstrated the application of *in silico* methodology for comparison of two different designs of two stent prototypes. Specifically, in [23], “the impact of strut thickness on mechanical characteristics of two different AB-BVS scaffolds” was analyzed: AB-BVS vs. AB-BVS-thinner, “as well as the impact of additional pocket holes (slots) in stent geometry on mechanical characteristics of two other types of Renuvia-PLLA stents”: PLLA-prot vs. PLLA-prot-slot. Numerical simulations were performed for radial compression, inflation, three-point bending, and two-plate crush resistance tests. It was proven that this methodology can be effectively applied to identify differences in effective stress distribution regarding changes in stent geometry and struct thickness. The results of the comparison also provided useful information about the zones of maximum stress, which is of great importance for stent analysis during the prototyping phase.

Another goal of the InSilc project was to develop and validate a mechanical modeling module, allowing *in silico* mimicking of all *in vitro* mechanical tests required by technical standards to assess a coronary drug-eluting BVS. In this paper, we present the implementation of this module using our in-house user interface (UI) software CAD Field and Solid, which allows the automatic generation and numerical analysis of the majority of the required ISO standard tests, as well as the postprocessing of the results. We also present the procedure for running *in silico* tests: local compression, tensile, kinking, and flex 1-3, which have been performed to compare the same designs of two stent prototypes: AB-BVS and Renuvia-PLLA, presented in [23]. As in [23], strut thickness and additional pocket slots in two different scaffolds are used as representative parameters for comparing the mechanical characteristics of the stents. The maximum stress value is also used as a measure of effectiveness and reliability of stent design.

## 2. Materials and Methods

The InSilc platform for *in silico* mechanical test validation is based on the integrated FE simulation and graphical interface software, PAK and CAD, respectively. PAK (abbreviation in Serbian of “Program za Analizu Konstrukcija”-“Program for Structural Analysis”) is high-performance finite element analysis (FEA) software, developed and implemented over decades at the University of Kragujevac and BioIRC (Bioengineering Research and Development Center, Kragujevac, Serbia) [24] for solving complex coupled multiphysics/multiscale problems, as well as contact problems. CAD Field and Solid (Figure 1(a)) is the in-house pre- and postprocessing 3D modeling and visualization tool developed at the University of Kragujevac and BioIRC using C++ programming language and the MFC (Microsoft Foundation Class) library. The CAD simplifies the model generation and can visualize and animate the results of computational simulations.

### 2.1. Component Architecture and Interoperability

The procedure for running FE simulations is divided into three steps: preprocessing, FE simulation, and postprocessing, Figure 1(b).

The CAD preprocessor is used for the generation of a model in a form that can be run using the FE simulation code PAK. To generate a model, it is necessary to choose several options in the CAD: a stent type, a test type, a material model for the stent and a test model, the time step, etc. The stent can be modeled using some external tool (ABAQUS) and exported to a mesh file with the extension ∗.inp. Optionally, the ∗.inp file is provided by the manufacturer. The mesh file consists of a list of the FE nodes and elements. The stent is then loaded into the CAD, and using the appropriate dialog, we can adjust parameters such as the stent position and orientation. The creation of the model usually consists of geometry and mesh generation, adding constraints, loads, and materials. Currently, the CAD has stents of various types in its database, from metal (Synergy) to bioresorbable (Absorb, Phantom Encore, or Renuvia) stents.

The FE model data containing a FE mesh and the aforementioned data are exported to a file with extension ∗.dat which is run by the FE solver PAK. The results of a FE simulation (field of displacement, velocities, pressures, concentrations, etc.) are exported to a file with extension ∗.unv that is automatically loaded by the postprocessor of the CAD. Additionally, results are exported in the form of ∗.vtk files that can be opened using Paraview visualization software. The file for postprocessing contains data about displacements, stress, and strains.

The CAD postprocessor is used for importing and visualization of the results and analysis by plotting various representations (field versus time, field within the space, etc.). Various options in the CAD offer to users to inspect the results per parameters.

### 2.2. Stent Designs

In this study, we use the same scaffolds that were used in [23], Figure 2. The first stent is a preproduction prototype supplied by Abbot, named absorb (AB-BVS), Figure 2(a). The manufacturer provided the same design with different thicknesses of the stent strut (AB-BVS-thinner), Figure 2(b). The second prototype is the Renuvia-PLLA supplied by Boston Scientific Limited. This prototype has the original geometry (PLLA-prot, Figures 2(c)) and the geometry with additional pocket slots (PLLA-prot-slots, Figures 2(d)). The FE mesh is modeled using isoparametric 8-node hexahedral elements, and data about stent designs is given in Table 1.

### 2.3. Computational Procedure

The problem is solved using the FE equations for solid mechanics, which is adequate for the representation of standard *in silico* mechanical tests. The displacement formulation is used, and the balance equation of a finite element is transformed into the implicit incremental-iterative form, and for iteration *i*, we have [25]

(1) $$\begin{array}{c} \left(\frac{1}{\Delta t^{2}}M+K\right)\Delta U^{\left(i\right)}=F^{\mathrm{ext}}-F^{\mathrm{int}\left(i-1\right)}-\frac{1}{\Delta t^{2}}M\left(U^{\left(i-1\right)}-U^{t}\right), \end{array}$$

where **U** and **U**^*t*^ are the nodal displacement at the previous iteration (*i* − 1) and at the start of a time step, respectively, **F**^ext^ are the external forces, and **F**^int(*i* − 1)^ are the internal forces according to the previous iteration (*i* − 1), while the matrices **M** and **K** are given in [25]. Iterations continue until the convergence criterion is satisfied.

The constitutive equations for a material model of poly-L-lactic acid (PLLA) stent are introduced in [22]. The material model uses direct experimental curves that are taken from the experiment. The experimentally recorded stress vs. strain relations are provided for three different strain rates at three different temperatures. The experimental stress-strain relation contains initial elastic behavior followed by a plastic zone. Using the interpolation procedure, it is possible from experimental curves to calculate equivalent stress ${\bar{\sigma }}^{\left(i-1\right)}={\bar{\sigma }}^{\left(i-1\right)}\left(e,\dot{e},T\right)$ as a function of current equivalent strain, equivalent strain rate, and temperature. Then, we calculate the final stress and factorize the tangent matrix. The steps we use for this purpose in our procedure for each iteration within one time step are [22] the following:

- Calculate equivalent stress ${\bar{\sigma }}^{\left(i-1\right)}$ and tangent constitutive matrix as *C*_*ij*_^*E*(*i* − 1)^, for the current equivalent strain ${\bar{e}}^{\left(i-1\right)}$ and equivalent strain rate ${\dot{\bar{e}}}^{\left(i-1\right)}$, using the tangent elastic modulus *E*_*T*_^(*i* − 1)^
- Calculate stress increments and stresses from the given curves as Δ*σ*_*k*_^(*i*)^ = *C*_*kj*_^*E*(*i* − 1)^Δ*e*_*j*_^(*i* − 1)^ and *σ*_*k*_^(*i*)^ = *σ*_*k*_^*t*^ + *C*_*kj*_^*E*(*i* − 1)^Δ*e*_*j*_^(*i* − 1)^, respectively
- Calculate ${\bar{\sigma }}_{\text{new}}^{\left(i-1\right)}$ from stresses and evaluate the stress ratio $r_{\text{stress}}={\bar{\sigma }}^{\left(i-1\right)}/{\bar{\sigma }}_{\text{new}}^{\left(i-1\right)}$
- Calculate final stresses as *σ*_*k*(final)_^(*i*)^ = *r*_stress_*σ*_*k*_^(*i*)^
- Factorize the tangent matrix as *C*_(final)*kj*_^*E*(*i* − 1)^ = *r*_stress_*C*_*kj*_^*E*(*i* − 1)^

Nonlinear contact between the stent and corresponding moving or static boundaries is modeled using the mechanism of two-body interaction presented in [26]. The contact is implemented using 1D elastic support elements that are generated every time the node of the moving boundary enters the finite element of the stent and is added to the system of linear equations for each time step until the end of the FE simulation. Within the CAD, the stiffness parameter of 1D contact elements can be defined. It is important to notice that excessive values can cause convergence problems, i.e., create a huge repulsive force between the stent and the moving or static boundary. The huge force will have an impulsive effect, and in a certain time step, there may be a big separation of the stent and the boundary, which will cause instability of the calculation and probably a failure of numerical simulation within that time step. In the case of a small stiffness parameter, a large penetration of one model into another (stent into the mold) can occur, which can lead to inadequate calculation solutions. The disadvantage of this procedure is that it usually takes several attempts until the user sets a value that leads to a successful FE calculation.

## 3. Results and Discussion

Four standard and general *in silico* tests, including the local compression, tensile, kinking, and flex 1-3 tests, are designed to test the stent's characteristics regarding its structural integrity through load/deformation characteristics. The material parameters of the stent are taken from [23].

### 3.1. Local Compression

The local compression test measures the deformation of the device in response to a localized compressive force [1, 27], the load required to permanently deform or fully collapse the stent, and determines whether the stent recovers its original geometry after the test. The *in vitro* test is usually performed on an axial load testing device at room temperature, where samples are immersed in pH 7.4 phosphate-buffered saline at 37°C for about 30 min [1] which mimics a clinically relevant environment, Figure 3(a).

In the *in vitro* test [1], the stent is positioned between the fixed plate and the trapped spike, Figure 3(b). The axial load testing device is compressing the stent at a trapped spike point, using the force which intends to compress the stent locally by at least half of its diameter. In the FE numerical simulation, the central stent axis is collinear with the *Z*-axis. Two rigid bodies are used for the fixed plate and the moving wedge (acting as a trapped spike), where the plate is collinear with the *XZ* plane while the central axis of the wedge lays in the *YZ* plane. The wedge is initially positioned at *y* = 1.69 mm, while the dimensions of the wedge and the bottom plate are shown in Table 2. The boundary condition used in the simulation is *u*_*x*_ = 0 for all stent nodes located in the *YZ* coordinate plane. The contact boundary condition according to [26] is set between stent outer surfaces and the plate surfaces. An axial displacement is applied via the wedge to mimic the use of appropriate localized compressive force. To ensure realistic *in vitro* conditions, the local compression FE simulation takes into account the residual displacements of the stent as a result of the inflation test, presented in [23], as well as obtained residual stresses.

The time period of the *in silico* simulation is 0.01 seconds while the prescribed displacement for the wedge is 1.8 mm, achieved in 100 time steps.  Figure 4 shows the results of the local compression test.

To measure the performance of two comparable designs, we are focused on the average stress distribution, as well as the maximum value of the stress, in the zones with the occurrence of the largest deformations. Smaller average stress distribution and smaller maximum stress will be a measure of better stent performance. From Figure 4, it can be seen that the AB-BVS-thinner model (Figure 4(b)) has achieved slightly better stress distribution compared to the original AB-BVS model (Figure 4(a)). This can especially be seen at the place where the wedge compressed the stent. On the other hand, the original PLLA-prot model (Figure 4(c)) achieved slightly better stress distribution compared to the PLLA-prot-slot model (Figure 4(d)). However, this “better” stress distribution of the PLLA-prot stent is insignificant since the stress has built up in the middle of the bridge of the PLLA-prot-slot stent instead of on the connection of the bridge and struts.

### 3.2. Tensile Test

The tensile test is the simplest experiment to characterize the mechanical response of coronary stents, particularly to assess the yield stress of the material. It is used to determine the longitudinal tensile strength of the struts, joints, and/or fixed connections of the stent device as a response to the longitudinal tensile load [1, 27]. The sample is fixed between specially designed fixtures, while the tensile load is applied in the longitudinal direction until the tested bond breaks or loses functional integrity, Figure 5(a).

In the FE simulation, the central stent axis is collinear with the *Z*-axis (Figure 5(b)). The nodes of two struts at the left side (bottom of the *Z*-axis) of the stent are constrained to move. The nodes of two struts at the right side (top of the *Z*-axis) of the stent are constrained in the *X* and *Y* directions, with applied prescribed displacement along the *Z*-axis. This test also takes into account the residual displacements and residual stresses obtained during the inflation test.

The time period of the *in silico* simulation is 1.01 seconds while displacement on the wedge of 3.6 mm is achieved through 100 steps. The results of the tensile test are shown in Figure 6.

In Figures 6(a) and 6(b), we can see that the results of the tensile test for the AB-BVS and AB-BVS-thinner stent model (Figures 6(a) and 6(b), respectively) are insignificantly different. However, the nonmodified model (AB-BVS stent) demonstrates slightly better stress distribution which can be observed at the connections between bridges and struts. Contrary to this, as for the results of the local compression test, the modified PLLA-prot-slot stent (Figure 6(d)) shows better results in the tensile test compared to the PLLA-prot stent (Figure 6(c)), which can be observed in connections between struts and bridges.

### 3.3. Kinking

Peripheral stents used in some anatomic locations will bend during normal body motion, such as knee flexion. The purpose of this test is to determine the minimum radius at which the deployed stent can be flexed without kinking or exhibiting a diameter reduction greater than 50%. The in vitro setup of the kinking test is shown in Figure 7(a).

In FE numerical simulation, the central stent axis is collinear with the *Z*-axis, Figure 7(b). Boundary condition *u*_*z*_ = 0 is applied to the nodes at the left end of the stent. The residual displacements and stresses, obtained by the radial compression test, presented in [23], are used here as an input. We are using simplified folding and unfolding for the balloon instead of using a full 3D balloon model. Therefore, the inflation of the stent is performed by using three deformable cylinders, within the initial diameter of 0.872 mm, while the length of each cylinder is 4.8 mm. These moving cylinders with a high stiffness are placed inside the stent and are used to simulate the balloon expansion. Displacements (*u*_1_, *u*_2_, and *u*_3_, Figure 7(b), top) are prescribed at the internal surface of the cylinders as a time-dependent function shown in Figure 8. A cylindrical shape mandrel (rigid body) is placed outside the stent, with three different diameters (1.5, 2.0, and 3 cm). The nonlinear contact 1D elements are used between the internal surfaces of the stent and the inner cylinder's outer surfaces and, second, between the outer stent surfaces and the inner stepwise surface of the outside cylindrical mandrel.

The time period of the *in silico* simulation is 0.031 seconds with 150 steps.

Figure 9 shows the results of the kinking test for all investigated cases. As it is shown in Figure 9, the AB-BVS-thinner model (Figure 9(b)) shows significantly better stress distribution compared to the AB-BVS model (Figure 9(a)). Similarly, the PLLA-prot-slot stent model demonstrates slightly better stress distribution than the PLLA-prot stent model (Figures 9(d) and 9(c), respectively).

### 3.4. Flex 1-3

In *in vitro* conditions, the flex test is performed by using the entire stent delivery system: a guide wire, catheter, and balloon. This delivery system is used to place the stent at the desired location inside the curved cylindrical mandrel. Then, the balloon is inflated, which expands the stent, and the stent rests on the inner surfaces of the mandrel. Finally, the balloon is deflated, and the entire delivery system is pulled out. Ideally, the stent remains attached to the inner surfaces of the cylindrical mandrel, Figure 10. In cases where the stent design is not satisfactory, malposition occurs with the stent, and that stent fails on the test.

Three different models of a flex mold were considered in this study: flex 1, flex 2, and flex 3, with diameters of the curve equal to 16, 20, and 24 mm, respectively. The dimensions of the flex 1 model are given in Figure 11(a), where the outer diameter of the curve is 20.7 mm which corresponds to 16 mm large median diameter. The models flex 2 and flex 3 are different in comparison to flex 1 regarding the value of diameter of the curvature, while the diameter of the pipe (3 mm) and the thickness of the mandrel (1 mm) remain the same. In the numerical simulation, the stent is initially positioned in a way that the central stent axis is collinear with the central axis of the inlet tube of the mandrel (Figure 11(b), *t*_0_). The curved cylindrical shape mandrel has characteristics of a rigid body. FE simulation is then performed by using the two-step procedure. In the first step, the stent is pulled in the direction of the mandrel by using the auxiliary 3D element and placed at the desired location (*t*_end_). In the second step, the surface pressures are prescribed at the internal surface of the stent, mimicking the balloon inflation and producing the stent expansion. The contact boundary condition is set between the outer stent surfaces and the inner surface of the cylindrical mandrel. The inputs to the model are the residual displacements and stresses, obtained as a result of the radial compression test. The geometrical setup of the flex tests is shown in Figure 11.

Two specific simplifications are introduced in the numerical model to provide the simulation of the described procedure in a reasonable time and with reasonable accuracy. First, we introduce a simplified procedure that does not include the use of a guide wire and a balloon. Instead, we use an auxiliary 8-node 3D element located in front of the stent which is connected to the upper side of the stent via its 4 nodes. Prescribed displacements (*u*_*e*_ and *u*_*i*_, Figure 11(b)) that are used to pull the stent are applied to the other four nodes of this auxiliary 8-node FE element. Using the appropriate algorithm, it is also ensured that this guide element always follows the axis of the cylindrical mandrel. Second, when the stent is brought to the appropriate position (final position, *t*_end_ at Figure 11(b)), i.e., when the central portion of the stent reaches the highest point of the mandrel, the auxiliary 8-node element stops moving, and the prescribed surface pressures begin to act on the inner surface of the stent, mimicking the balloon expansion. An illustration of the stent before (dashed red line) and after the expansion (full blue line) is given in Figure 11(b).

Figures 12 and 13 show the results of the flex 1 test for all stent models. It can be observed that the nonmodified model of the AB-BVS stent (Figure 12(a)) shows significantly better stress distribution than the modified AB-BVS-thinner stent model (Figure 12(b)). Similarly, the modified PLLA-prot-slot stent model demonstrates better stress distribution in comparison to the nonmodified PLLA-prot stent model (Figures 13(b) and 13(a), respectively).

Figures 14 and 15 show the results for the flex 2 test. It can be observed that, unlike in the flex 1 test, the AB-BVS-thinner stent model shows significantly better stress distribution than the AB-BVS stent model (Figures 14(b) and 14(a), respectively). Likewise, the PLLA-prot-slot model shows better stress distribution than the PLLA-prot stent model (Figures 15(b) and 15(a), respectively).

Figures 16 and 17 show the results of the flex 3 test for all stent models. As can be observed in Figure 16, the results of the flex 3 test are very similar for AB-BVS and AB-BVS-thinner stent models (Figures 16(a) and 16(b), respectively). The stress distribution is slightly better on the AB-BVS-thinner model. The PLLA-prot stent model shows better stress distribution compared to the PLLA-prot-slot stent model (Figures 17(a) and 17(b), respectively), though it is not fully inflated.

## 4. Discussion

In this paper, a computational tool integrated into the InSilc platform for testing biodegradable stents is presented. There are two versions of the InSilc stent test tool. The first is the one that has been converted into a console application available on the cloud platform and integrated within the official protocol (https://insilc-front.herokuapp.com/). The second version is Windows-based and allows users to prescribe geometry and perform one of the tests following the user interface on the Windows platform (https://github.com/miljanmilos/CAD-Solid-Field). The integrated tool can be used for any input geometry. Preparing an example using our graphical interface is very easy and simple. Setting constraints, materials, and contact takes several hours, which also stands for running a numerical simulation for simple geometric models with less than 100,000 FE mesh nodes. Visualization of the results is available in the postprocessing tool. It is also possible to export the results to a file with the extension ∗.vtk and visualize the results using modern software (e.g., Paraview).

Simulations of mechanical tests are performed on two different types of stents: AB-BVS and PLLA. These two prototypes were of special interest for the recently completed InSilc project (http://www.insilc.eu), for which it was necessary to provide an estimation of mechanical stresses and to help in the decision of whether those prototypes have the potential to enter the production phase. Since both prototypes are intended to be made of biodegradable polymer with low stiffness, strain rate sensitivity, and plastic behavior, it was a challenge to propose an adequate modeling and simulation strategy. It is also a challenge to run *in silico* simulations that are a simplified version of the real mechanical test and to provide reliable conclusions regarding the type and geometry of the scaffold.

Two factors were of the main interest for the analysis presented in this work: the effect of struct thickness in the AB-BVS prototype and the effect of additional slots within the stent geometry of the PLLA prototype. The results of the local compression test (Figures 4(a) and 4(b)), noticed at the place where the wedge compressed the stent, show better stress distribution in the AB-BVS-thinner model compared to the standard AB-BVS model. The same test for the PLLA prototype (Figures 4(c) and 4(d)) shows better stress distribution within the PLLA prototype in comparison to the PLLA prototype with additional slots. The results of the tensile test (Figure 6) showed that there were no significant differences between effective stresses for the AB-BVS and AB-BVS-thinner prototypes. By observing connections between struts and bridges, the AB-BVS stent showed smaller stresses in comparison to the thinner model, while the PLLA prototype with slots showed better results compared to the standard PLLA prototype. The result of the kinking test (Figure 9) suggests that the AB-BVS-thinner had better performance in comparison to the original AB-BVS model, while the standard PLLA prototype achieved lower stresses compared to the PLLA prototype with slots. The flex test showed different results when using flex 1, 2, and 3. For flex 1, the AB-BVS stent showed significantly better stress distribution than the modified AB-BVS-thinner stent model. Similarly, the modified PLLA prototype with slots displayed better results than the standard PLLA model. Opposite results were obtained for the flex 2 and AB-BVS prototypes, but the PLLA prototypes showed the same behavior as flex 1. Finally, the flex 3 test showed a slightly better stress distribution in the thinner model, while the PLLA-prot stent model had better results in stress distribution compared to the PLLA prototype with slots.

Some simplifications in relation to the realistic kinking and flex mechanical tests were made in the numerical model. In the kinking test, we used three deformable cylinders to simulate the balloon expansion. By prescribed displacement applied to each of the cylinders, it was possible to inflate the cylinders and expand the stent. In the flex test, we used an auxiliary 3D element instead of the guide wire. The use of guide wire would lead to additional FE elements which would slow down the numerical simulation. In this case, it would be also necessary to model the nonlinear contact between the wire and the balloon, as well as between the wire and the stent, using the procedure described in [26]. Second, when the stent was positioned at the desired place within the curved mandrel, we used prescribed surface pressure instead of full 3D balloon inflation, since the use of a full balloon model would introduce additional assumptions into the model. Namely, the balloon itself would have to be modeled, which would lead to an additional number of finite elements. Also, the balloon should be implemented either as a shell or as a 3D element, and additional contact elements between the balloon and the stent. It would also lead to additional equations in the FE simulation, but probably also to additional problems we would have to face during the release of numerical simulations.

A limitation of the study is that the computational tool still does not provide a simulation procedure for the two remaining ISO standard tests. These are the radial fatigue test (i.e., deployment of the implantation system within a deformable tube, where the cyclic pressure is imposed in the tube with deployed stent), and the S tube test (i.e., the stent is moved within a properly curved rigid tube). Additionally, there is no demonstration regarding the change in radial force, since this is one of the conclusive parameters bearing in mind the possibility of stent collapse in contact with stenosis. By addressing those issues, we believe that this kind of integrated software has the potential to become a validation and optimization tool for different types of PLLA-based stent prototypes.

## 5. Conclusions

In this research, we presented the capabilities of a validated numerical model to simulate the mechanical behavior of preproduction stent prototypes. The material model used for the FE analysis is based on experimental curves and offers the possibility to use any experimentally recorded constitutive curve of the stent material as an input. The integrated InSilc test tool simplifies model generation and prototype testing and can be potentially used for any bioresorbable prototype scaffold. These *in silico* tests can reduce the need for mechanical tests, as well as reduce the cost of the design process itself. They also ensure that at an early stage, after the application of the tests, a decision can be made whether or not the stent prototype should enter the redesign phase. Stress distribution solutions, provided by the software, can be of great help in comparing two or more prototypes and can help researchers to decide whether a proposed design has the potential to be produced and to enter the real mechanical tests.

In this paper, we demonstrated numerical simulations (local compression, tensile test, kinking, and flex) of mechanical tests requested by appropriate ISO standards for testing stent devices. For all the aforementioned tests, we provided detailed descriptions and challenges on the path for successful simulation runs in a reasonable time, with acceptable accuracy according to applied simplifications. It was shown that strut thickness and additional pocket holes (slots) are the parameters that can significantly change the distribution of the stresses and the maximum stress values for the AB-BVS and PLLA-prot stent prototypes.

The computational tool presented in this paper can be further improved to include the deployment of the implantation system within a deformable tube, where the cyclic pressure is imposed in the tube with a deployed stent, and also the analysis of radial force change. By including these aspects in the computational platform, this software has the potential to serve as a stent prototype validation and optimization tool.

## Figures and Tables

**Figure 1:** (a) CAD field and solid graphical pre- and postprocessing user interface software (https://github.com/miljanmilos/CAD-Solid-Field); (b) data flow: software scheme for input/output data.

**Figure 2:** Stent geometries with the region of interest: (a) AB-BVS stent; (b) AB-BVS-thinner stent; (c) PLLA-prot stent; (d) PLLA-prot-slot stent.

**Figure 3:** (a) Real mechanical test setup for local compression test [1]; (b) geometrical setup and boundary conditions for FE numerical simulation of local compression test.

**Figure 4:** Results for local compression test: (a) AB-BVS stent, (b) AB-BVS-thinner, (c) PLLA-prot, and (d) PLLA-prot-slots.

**Figure 5:** (a) Real mechanical test setup for longitudinal tensile test [1]; (b) geometrical setup and boundary conditions for FE numerical simulation of tensile test.

**Figure 6:** Results for tensile test of (a) AB-BVS stent, (b) AB-BVS-thinner, (c) PLLA-prot, and (d) PLLA-prot-slots.

**Figure 7:** (a) Real mechanical test setup for kinking test [1]; (b) geometrical setup and boundary conditions for FE numerical simulation for kinking test; dimensions are given in mm.

**Figure 8:** Function of displacements for each cylinder in kinking test, according to Figure 7(b)—*u*_1_ (left cylinder), *u*_2_ (middle cylinder), and *u*_3_ (right cylinder).

**Figure 9:** Results for kinking test: (a) AB-BVS stent, (b) AB-BVS thinner, (c) PLLA-prot, and (d) PLLA-prot-slots.

**Figure 10:** Real mechanical test setup for flex test for three different configurations with diameters of the flex curve of *d* = 24, 20, and 16 mm.

**Figure 11:** (a) Geometrical characteristics and (b) simulation protocol for flex 1 test.

**Figure 12:** Results for flex 1 test of (a) AB-BVS stent and (b) AB-BVS-thinner.

**Figure 13:** Results for flex 1 test of (a) PLLA-prot and (b) PLLA-prot-slots.

**Figure 14:** Results for flex 2 test of (a) AB-BVS and (b) AB-BVS-thinner stent model.

**Figure 15:** Results for flex 2 test of (a) PLLA-prot and (b) PLLA-prot-slot stent model.

**Figure 16:** Results for flex 3 test: (a) AB-BVS stent and (b) AB-BVS-thinner.

**Figure 17:** Results for flex 3 test of (a) PLLA-prot and (b) PLLA-prot-slots.

**Table 1:** Data about geometry and FE mesh for scaffolds used in our study.

Sent name	AB-BVS	AB-BVS-thinner	PLLA-prot	PLLA-prot-slots
Outer radius (mm)	1.65	1.62	1.62	1.62
Inner radius (mm)	1.49	1.49	1.5	1.5
Length (mm)	12.18	12.18	15.68	15.68
No. of hexahedral FE elements	46728	46728	49488	40908

**Table 2:** Geometrical characteristics of plates used in local compression test.

Plate	Height (mm)	Width (mm)	Depth (mm)
Wedge	2.2	0.6	0.6
Bottom plate	0.2	30.4	4

## Data Availability

The online version of the InSilc platform is available at https://insilc-front.herokuapp.com/login (credentials required). The executable of the CAD Solid and Field, used as interface software for local pre- and postprocessing on Windows OS, has been deposited in the GitHub repository https://github.com/miljanmilos/CAD-Solid-Field.
